The article "Patellar Height after High Tibial Osteotomy of the Distal Tibial Tuberosity: A Retrospective Study of Age Stratification" was published in 2022. Journal: Comput Math Methods Med.

# Patellar Height after High Tibial Osteotomy of the Distal Tibial Tuberosity: A Retrospective Study of Age Stratification

**DOI:** 10.1155/2022/7193902

**Published:** 2022-01-27

**Authors:** Tiansong Ding, Yetong Tan, Xiangdong Tian, Zhipeng Xue, Sheng Ma, Yuanyi Hu, Ye Huang, Xiaomin Li

**Affiliations:** ^1^Beijing University of Chinese Medicine, Beijing 100029, China; ^2^Minimal Invasive Joint Department, The Third Affiliated Hospital of Beijing University of Chinese Medicine, No. 51 Anwai Xiaoguan Street, Chaoyang District, Beijing 100029, China

## Abstract

**Objective:**

To explore the effect of age stratification on patellar height after single-plane high tibial osteotomy of the distal tibial tuberosity (DTT-HTO).

**Methods:**

A retrospective analysis was performed on 110 knee joints undergoing DTT-HTO. Patients were divided into three groups according to age: under 60 years old, 28 cases; 60 to 70 years old, 61 cases; and over 70 years old, 21 cases. All patients were followed up for no less than 12 months, and at each follow-up, short-leg radiographs and whole-leg radiographs were taken. The values of the Caton-Deschamps index (CDI) and Blackburne-Peel index (BPI) of single-short-leg radiographs and the femoral-tibial angle (FTA) and weight-bearing line ratio (WBLR) of whole-leg radiographs were measured before and at the last follow-up. The Lysholm score before and at the last follow-up and the visual analogue scale (VAS) score before and 3 days after surgery and at the last follow-up were calculated. The frequency of classification of the normal-height patella, patella alta, and patella baja before and after surgery was recorded.

**Results:**

There were no significant differences in CDI and BPI preoperatively or postoperatively among the three groups (*P* > 0.05), and there were no statistically significant differences in FTA and WBLR. There were no significant differences in CDI, BPI, FTA, or WBLR between the three groups before and after the operation (*P* > 0.05). The Lysholm score increased from 48.84 ± 10.10 before surgery to 91.96 ± 3.082 after surgery (*P* < 0.05); the VAS score decreased from 8.23 ± 0.99 before surgery to 1.93 ± 0.953 at 3 days after surgery and 1.07 ± 0.53 at the last follow-up (*P* < 0.01). No significant difference was observed in the incidence of each patellar height classification between the three groups preoperatively and postoperatively.

**Conclusion:**

Patellar height is not influenced by DTT-HTO. The age of patients is not a limiting factor for the selection of this surgical procedure. Without affecting the height of the patella, DTT-HTO can effectively reduce pain in the knee joint, restore the function of the knee joint, and delay the progression of patellar arthritis.

## 1. Introduction

High tibial osteotomy is one of the surgical methods for treating medial compartment knee osteoarthritis. Traditional HTO is divided into closing-wedge high tibial osteotomy (CWHTO) and open-wedge high tibial osteotomy (OWHTO), and both procedures can effectively correct the coronal weight-bearing line of the knee joint, transfer the lower limb alignment from the medial compartment of the knee joint to the lateral compartment, increase the stress area of the tibiofemoral joint, and reduce the pressure of the medial compartment to relieve medial compartment knee pain and help patients recover walking function [1–13]. The mechanical properties of a biostructure depend on its Young's modulus (*E*). Therefore, it is likely that a harder substance has a larger *E* [14]. For instance, the value of *E* for bone is 14 GPa. However, HTO can also affect the postoperative bone structure of the patellofemoral joint, resulting in patella alta or patella baja compared to the preoperative situation. Therefore, measurement methods [15] such as CDI [16] and BPI [16] are often used to test whether the height of the patella changes.

There are different opinions about the effect of HTO on patellar height, but a consensus has already been reached regarding whether high tibial osteotomy above the tibial tuberosity can affect patellar height [6, 12, 17–20]. This was confirmed by previous retrospective clinical studies of DTT-HTO conducted by our team [9]. Patellar height disorder can lead to cartilage degeneration of the patellofemoral joint, loss of function, knee pain, and recurrent patellofemoral dislocation. The pressure on the patellofemoral joint increases during the bending of the patella baja; therefore, the possibility of patellofemoral joint degeneration increases [2]. Patellar instability is often associated with patellar alta, and long-term patellar instability can lead to knee pain, functional limitations, and osteoarthritis. The inability causes the patella to move outward when knee flexural activity, especially during the first 30°, is unable to pull the patella [21]. Because of the patella alta state, the contact area between the patella and the femur decreases, the pressure increases, and the patellofemoral joint wear increases, resulting in patellofemoral chondromalacia [22].

Current literature reports that HTO is suitable for young, active knee osteoarthritis patients with high functional needs. In previous studies, 60 years [23–25] or 65 years [26] was the age limit often used as the inclusion criterion for HTO surgical indicators. This may be due to the influence of certain variables (such as osteoporosis) that change with age on the outcome of surgery. However, it has been found that a number of knee osteoarthritis (KOA) patients aged over 60 or 65 years old also achieve good clinical efficacy by HTO in clinical practice. They often experience relief from knee pain in a short period of time and gradually recover walking, going up and down the stairs, flexion and extension functions, and so on. More research on the effect of HTO on patellar height has focused on the choice of surgical procedures; some studies have challenged the age limitation in HTO inclusion criteria, but no literature has been found on the effect of age on patellar height after HTO. The purpose of this study was to observe the influence of age on patellar height after DTT-HTO and to explore whether the age restriction can be broken and whether more surgical options can be provided to patients with KOA.

## 2. Methods

### 2.1. Patients

A retrospective study of 128 patients who received DTT-HTO in the Third Affiliated Hospital of Beijing University of Chinese Medicine from August 2016 to June 2020 was conducted. Except for the 18 cases that were removed according to the inclusion and exclusion criteria, a total of 110 patients aged 51 to 82 were divided into three groups according to age: under 60 years old, 28 cases; 60 to 70 years old, 61 cases; and over 70 years old, 21 cases. There was no significant difference in demographics or parameters among the three groups (Table 1). Inclusion criteria are as follows: (1) medial compartment arthritis of grade k-L: ≥3, lateral: ≤1; (2) follow-up time ≥ 12 months; and (3) image data that were completed and that comprised approximately 30° flexion knee lateral radiographs and whole-leg radiographs before and at the last follow-up. Exclusion criteria are as follows: (1) rotational angles existing between the medial femoral condyle and the lateral femoral condyle in one of the lateral radiographs and (2) patients suffering from types of arthritis other than KOA.

### 2.2. Operative Procedure

Starting from 1 cm below the midpoint of the medial joint line, an incision of approximately 5 cm was made downward to separate the skin, subcutaneous, deep fascia, muscle, and periosteum in turn to expose the tibial bone surface (Figure 1(a)), avoiding harming the patellar tendon and pes anserinus. A Kirschner wire was inserted from the distal tibial tubercle to 0~1 cm below the tibiofibular fornix at an angle of 30° to 45° to the vertical line of the longitudinal axis of the tibia. The position of the Kirschner wire was observed on the C-arm, and a bone saw cut the medial tibia off along the Kirschner wire (Figure 1(b)), leaving 1 cm of cortical bone on the lateral side of the tibia. The lateral cortex was loosened by drilling holes from the osteotomy area to the lateral residual cortex (Figure 1(c)). The assistant performed valgus and rotation stress on the operative limb, and the surgeon used a bone knife to open it up (Figure 1(d)) to change the lower limb alignment. C-arm fluoroscopy showed that the WBL passed lateral to the lateral tibial intercondylar eminence at the Fujisawa point. Bone substitutes were implanted (Figure 1(e)), a guide plate and screws were inserted (Figure 1(f)), and the wound was finally sewn up.

Ankle pump exercises were performed in bed on the first day after surgery, and patients were allowed to step on the ground with the aid of a walker on the third postoperative day. The patients advanced to walking with two crutches two weeks after the surgery and with a single crutch four weeks after the surgery. Walking without auxiliary devices was achieved 8 to 12 weeks after the surgery.

### 2.3. Radiological Measurements

All patients were photographed before surgery and at the last follow-up to observe the fixation of the guide plate and screws and the changes in CDI, BPI, FTA, and WBLR. All images were taken by the same technician and the same machine (GE Definium 6000 DR) and were independently measured by two project team members.

The Caton-Deschamps index is the ratio between the length from the lowest point of the patellar articular surface to the anterior tip of the tibial tuberosity and the patellar joint surface (*B*/*A*). BPI is the ratio of the vertical distance from the lowest point of the patellar articular surface to the medial tibial plateau line (*D*) to the patellar articular surface (*C*/*A*). FTA is the angle (*α*) formed by the anatomical axis of the femur (*F*) and tibia (*G*) at the center of the knee joint (Figure 2). WBLR is the distance from the intersection of the lower limb alignment and the tibial plateau to the medial edge of the tibial plateau (*H*) divided by the width of the tibial plateau (*I*) (Figure 3). The CDI and BPI were measured on lateral radiographs in mild degrees of flexion (30°). FTA and WBLR were gauged on non-weight-bearing lateral radiographs.

### 2.4. Clinical Evaluation

The Lysholm score was used to assess the knee status before and at the last follow-up, including gait, function, pain, swelling, and stability. The visual analogue scale (VAS) was used to assess the degree of pain before and 3 days after surgery and at the last follow-up, with a score ranging from 0 to 10. The frequencies of the normal-height patella, high patella, and low patella in the three groups were compared before and after the operation.

### 2.5. Statistical Analysis

All the collected data were analyzed using SPSS (version 25.0; SPSS, China). A paired *t*-test was used to analyze the CDI, BPI, FTA, and WBLR in the groups. Single-sample analysis of variance was used between the groups. A paired *t*-test was used to compare the preoperative and postoperative Lysholm scores, and repeated-measure ANOVA was used to detect the changes in VAS scores before surgery, 3 days after surgery, and at the last follow-up. The chi-square test was used to compare the changes in patellar height classification in the three groups before and after surgery.

## 3. Results

There were no significant differences in CDI and BPI preoperatively or postoperatively among the three groups (*P* > 0.05), and the differences in FTA and WBLR were statistically significant (*P* < 0.05). No significant differences were observed in CDI, BPI, FTA, or WBLR between the three groups before and after surgery (*P* > 0.05) (Table 2).

The Lysholm score of the knees increased from 48.84 ± 10.10 before the operation to 91.96 ± 3.082 at the last follow-up (*P* < 0.05). The VAS score decreased from 8.23 ± 0.99 before surgery to 1.93 ± 0.953 on the third postoperative day and 1.07 ± 0.53 at the last follow-up (*P* < 0.01) (Table 3).

The incidences of the normal patella, patella alta, and patella baja (CDI < 0.8 was taken as the standard) were 53.57%, 17.86%, and 28.57%, respectively, in the <60-year-old group before surgery and 50.00%, 17.86%, and 32.14%, respectively, at the last follow-up. The incidences of the three types of patellar heights in the 60~70-year-old group were 52.50%, 14.75%, and 32.79%, respectively, before surgery and 47.54%, 14.75%, and 37.70%, respectively, at the last follow-up. The incidences of the three types of patellar heights before surgery in the >70-year-old group were 52.50%, 14.75%, and 32.79%, and these incidences were 47.54%, 14.75%, and 37.70%, respectively, at the last follow-up. There were no significant differences among the three groups preoperatively and postoperatively (Table 4).

One patient in the <60-year-old group, five patients in the 60~70-year-old group, and one patient in the >70-year-old group had a suspicious low patella after knee surgery (0.6 < CDI < 0.8). Decreases in patellar height were not observed after surgery in the three groups (CDI < 0.6) (Table 5).

## 4. Discussion

### 4.1. Influence of HTO on Patellar Height in Previous Literature

CWHTO has a long history. Disadvantages of bone mass on the tibiofibular joint and the risk of common fibular nerve injury have caused it to be surpassed by OWHTO, which can avoid these problems and control the osteotomy angle and WBL more accurately and easily; however, bone substitutes are needed, and the healing speed declines in the osteotomy area because of cortical bone [4]. The patellar tendon is the lower part of the quadriceps femoris muscle, starting from the lower margin of the patella and ending at the tuberosity of the tibia [27]. Classical OWHTO was performed through the superior tibial tuberosity. Expansion of the osteotomy area resulted in the distal displacement of the tibial tuberosity and increased tensile stress of the patellar tendon, which pulled the patella to the distal end of the limb and led to changes in the height of the patella [5]. On this basis, the greater the osteotomy angle, the more obvious the patellar height decrease [13]. Contracture of the patellar tendon after osteotomy may also result in a decrease in the height of the patella [28].

CWHTO avoids osteotomy above the tibial tuberosity. In the meta-analysis of 28 trials included by Cheng et al. [29], no significant change in patellar height was seen after CWHTO. Tigani et al. [6] measured the patellar height after OWHTO and CWHTO by CDI and found that the patellar height of OWHTO decreased more significantly during at least 1 year of postoperative follow-up. Even in OWHTO, biplanar descending OWHTO (osteotomy line at the distal tibial tuberosity) did not affect patellar height compared with biplanar ascending OWHTO (osteotomy line at the proximal tibial tuberosity) [7]. Warner et al. [5] performed subtubercle osteotomy in the treatment of MCOA combined with the Ilizarov technique. They found that the height of the patella (CDI) in 72 knees did not change significantly after the operation and that the patellofemoral relationship was normal. Next, Bayam et al. [8] combined STO with the fixator-assisted nailing technique to perform orthopedic procedures on 32 knee joints, and the study confirmed that the patellar height was not affected during at least 30 months of follow-up. In a large number of clinical studies, it has been confirmed that whether the osteotomy line passes through the tibial tuberosity is one of the evaluation criteria for the change in patellar height, and subtubercle osteotomy can effectively avoid this [3–5, 7–12].

Some studies [2] have shown that open-wedge proximal tibial osteotomy can significantly increase the pressure on the patellofemoral articular cartilage at 30°, 60°, and 90° knee flexion and accelerate the degeneration of the patellofemoral articular cartilage. Sim et al. [30] found that patellar height decreased after OWHTO, and single-photon emission computed tomography and conventional computed tomography (SPECT/CT) were used to capture the contact stress of the patellofemoral joint. The results showed that the contact stress increased in 7.1% of the knees, the articular cartilage of the patella and femoral trochlea significantly deteriorated, and the grade of patellofemoral arthritis was elevated.

### 4.2. Influence of Age on Radiological and Clinical Outcomes after HTO

Although some studies on HTO have included age as a criterion, it should not be used as a mandatory screening criterion for the treatment of older KOA patients. One study found that radiological outcomes in patients receiving OWHTO were not affected by age, and clinical outcomes (HSS, KSS) were affected by cartilage status rather than age per se [31]. Kuwashima et al. [32] found that, compared with the preoperative KSS score, only the functional activity score showed differences in the group aged ≥65 years and ≤64 years, while differences in the symptom score, satisfaction score, and expectation score were not statistically significant. Kohn et al. [33] found that the improvement of pain symptoms (VAS score) and functional status (Lysholm score) of knees after HTO showed no significant difference between the young group and the old group. They believed that the postoperative efficacy of HTO patients was determined not by their age but by the state of knee soft tissue. Goshima et al. [34] divided OWHTO patients into two groups, older than 65 years old and younger than 65 years old, and conducted follow-up for up to 24 months. It was concluded that age did not affect the clinical and imaging results after HTO. To enhance the medical image analysis, superresolution image enhancement of the medical scans may be applied based on techniques such as deep learning [35].

### 4.3. The Effect of DTT-HTO on Patellar Height in This Study

DTT-HTO was simple to perform and effectively avoided patellar lowering or elevation. Seven of 110 knee joints decreased from the normal-height patella (0.8 < CDI < 1.2) to the low patella (CDI < 0.8) in the image measurement data, but the overall height of the patella was not affected (*P* > 0.05), which may be related to measurement errors. The authors reviewed the factors affecting patellar height, including knee function, scarring on the patellar ligament, contracture [28], and the motion of the quadriceps femoris [12, 36]. Therefore, preoperative protection of the knee joint, avoidance of accidental injury of the patellar ligament during the operation, and postoperative rehabilitation exercise can contribute to the recovery of knee joint function. Other various algorithms can be used to improve medical imaging procedures [37]. The bone structure integrity is heavily influenced by the material properties that are dependent on certain characteristics [38, 39].

### 4.4. Relationship of Patellar Height to Osteoporosis

Aging is one of the predisposing factors of osteoporosis; current international literature mainly considers the group aged >60 or 65 years as the high-risk population of osteoporosis [40]. Other operations of HTO, such as OWHTO, performed osteotomy above the tibial tuberosity, where there is abundant cancellous bone. Affected by the position of the osteotomy line, the supporting stress of internal fixation was mainly concentrated above the tibial tuberosity. If the patient with KOA also has osteoporosis, the screws, inserted to fix the guide, have the potential to cut cancellous bone under body gravity, resulting in bone loss and biomechanical environment disorder in the patellofemoral joint. DTT-HTO can avoid this happening effectively.

### 4.5. Limitation

The limitations of our study are as follows. (1) The short follow-up time made it impossible to explore the long-term effect of DTT-HTO on patellar height. (2) The observation indicators mainly focused on the image measurement method, and the results had errors. (3) Other factors contributing to the changes in body mechanisms associated with aging have not been explored more broadly. (4) The influence of osteoporosis on HTO has not been further studied.

## 5. Conclusion

DTT-HTO did not change the height of the patella at different ages, WBL and FTA were corrected, pain was relieved, and function was recovered. Based on the clinical trial results of this study, patients should not be forced to give up their choice of HTO simply because of their age. We recommend that the inclusion criteria for HTO be improved to provide more surgical options and benefit elderly KOA patients.

## Figures and Tables

**Figure 1:** Intraoperative operation of DTT-HTO. (a) Exposure of the tibial bone surface. (b) The medial tibia was sawed by a bone saw along the Kirschner wire route. (c) Use of a Kirschner wire to drill holes from the osteotomy area to the opposite side to weaken the lateral bone cortex. (d) Opening up the osteotomy area with the bone knife. (e) Implantation of bone substitutes. (f) Placement of the guide plate and its fixation with screws.

**Figure 2:** Methods of image measurement. (a) CDI = *B*/*A*. (b) BPI = *C*/*A*. (c) FTA = *α*.

**Figure 3:** Method of WBL. (a) WBLR_1_ = *H*_1_/*I*_1_. (b) WBLR_2_ = *H*_2_/*I*_2_.

**Table 1:** Characteristics of the three groups.

	<60 years (*n* = 28)	60~70 years (*n* = 61)	>70 years (*n* = 21)	Value	*P*
Sex					
Male	8	15	5	*χ* ^2^ = 0.197	0.906
Female	20	46	16		
Knee					
Left	20	33	15	*χ* ^2^ = 3.458	0.178
Right	8	28	6		
Duration of disease (years)	8.50 ± 1.972	8.85 ± 2.056	9.29 ± 2.935	*F* = 0.747	0.476
BMI (body mass index) (kg/m^2^)	26.40 ± 3.046	26.38 ± 3.195	25.89 ± 2.586	*F* = 0.224	0.800
BMD *t*-score					
≤-2.5 (%)	2	9	6	*χ* ^2^ = 5.508	0.239
>-2.5~≤-1.5 (%)	5	15	6		
>-1.5 (%)	19	37	9		
Varus deformity (°)	8.71 ± 2.088	9.16 ± 2.099	9.62 ± 2.519	*F* = 1.043	0.356
Duration of follow-up (months)	20.86 ± 5.707	21.64 ± 4.401	24.05 ± 4.78	*F* = 2.815	0.064

**Table 2:** Changes in imaging indicators in the three groups ($\bar{x}\pm s$).

	Groups	Preoperative	Postoperative	*t*	*P*
CDI	<60 years	0.88 ± 0.11	0.88 ± 0.121	-0.113	0.911
	60~70 years	0.87 ± 0.15	0.85 ± 0.156	1.569	0.122
	>70 years	0.90 ± 0.132	0.89 ± 0.131	1.333	0.197
*F*		0.422	0.537		
*P*		0.657	0.586		
BPI	<60 years	0.85 ± 0.124	0.87 ± 0.126	-0.854	0.401
	60~70 years	0.89 ± 0.128	0.88 ± 0.131	1.986	0.052
	>70 years	0.90 ± 0.08	0.91 ± 0.071	-0.285	0.779
*F*		1.256	0.812		
*P*		0.289	0.447		
WBLR	<60 years	0.18 ± 0.084	0.55 ± 0.089	-23.184	<0.01
	60~70 years	0.18 ± 0.138	0.59 ± 0.10	-20.136	<0.01
	>70 years	0.19 ± 0.089	0.61 ± 0.041	-19.481	<0.01
*F*		0.029	0.713		
*P*		0.972	0.492		
FTA	<60 years	182.96 ± 2.063	172.39 ± 3.919	15.884	<0.01
	60~70 years	183.57 ± 2.171	171.02 ± 3.359	25.800	<0.01
	>70 years	183.48 ± 2.112	170.62 ± 2.459	18.605	<0.01
*F*		0.830	2.046		
*P*		0.439	0.134		

**Table 3:** Preoperative and postoperative score changes of the affected knee ($\bar{x}\pm s$).

	Preoperative	Third postoperative day	Last follow-up	Value	*P*
Lysholm	48.84 ± 10.10	—	91.96 ± 3.082	*t* = −36.662	<0.01
VAS	8.23 ± 0.99	1.93 ± 0.953	1.07 ± 0.53	*F* = 1461.907	<0.01

**Table 4:** Changes in the frequency of patellar height classification (*n* = 110, %).

		Normal patella	Patella alta	Patella baja	*χ* ^2^	*P*
<60 years	Preoperative	15 (53.57)	5 (17.86)	8 (28.57)	0.093	0.954
	Postoperative	14 (50.00)	5 (17.86)	9 (32.14)		
60~70 years	Preoperative	32 (52.50)	9 (14.75)	20 (32.79)	0.357	0.837
	Postoperative	29 (47.54)	9 (14.75)	23 (37.70)		
>70 years	Preoperative	11 (52.38)	5 (23.81)	5 (23.81)	0.155	0.926
	Postoperative	12 (57.14)	5 (23.81)	4 (19.05)		

**Table 5:** Outcomes of patellar height in the three groups (*n* = 110, cases).

	Preoperative	Postoperative	
<60 years	Normal patella	Normal patella	
		+	-
	+	14	1
	-	0	13
	Patella alta	Patella alta	
		+	-
	+	5	0
	-	0	23
	Patella baja	Patella baja	
		+	-
	+	8	0
	-	1	19
60~70 years	Normal patella	Normal patella	
		+	-
	+	27	5
	-	2	27
	Patella alta	Patella alta	
		+	-
	+	9	0
	-	0	52
	Patella baja	Patella baja	
		+	-
	+	18	2
	-	5	36
>70 years	Normal patella	Normal patella	
		+	-
	+	10	1
	-	2	8
	Patella alta	Patella alta	
		+	-
	+	5	0
	-	0	16
	Patella baja	Patella baja	
		+	-
	+	3	2
	-	1	15

## Data Availability

Data are available on request from the authors due to privacy/ethical restrictions.

## Abbreviations

KOA: Knee osteoarthritis
DTT-HTO: Distal tibial tuberosity high tibial osteotomy
CDI: Caton-Deschamps index
BPI: Blackburne-Peel index
VAS: Visual analogue scale
FTA: Femoral-tibial angle
WBLR: Weight-bearing line ratio
CWHTO: Closing-wedge high tibial osteotomy
OWHTO: Open-wedge high tibial osteotomy.
